The article "Study on 3D Image Reconstruction Model of Sparring Action Based on Graph Neural Network (GNN)" was published in 2021. Journal: Comput Intell Neurosci.

# Study on 3D Image Reconstruction Model of Sparring Action Based on Graph Neural Network (GNN)

**DOI:** 10.1155/2021/6882467

**Published:** 2021-10-27

**Authors:** Yahui Chang, Meng Su

**Affiliations:** ^1^School of Physical Education, ShanXi University, Taiyuan 030006, Shanxi Province, China; ^2^Department of Physical Education, The Graduate School of Dankook University, Yongin-si 16890, Gyeonggi-do, Republic of Korea

## Abstract

With the advent of the information age, human demand for information is increasing day by day. The emergence of the concept of big data has triggered a new round of technological revolution, and visual information plays an important role in information. In order to obtain a better 3D model, this paper studies the reconstruction model of training motion 3D images based on a graphical neural network algorithm. This paper studies the problem of Sanda from the following two aspects. First, we try to apply two deep learning algorithms, graphical neural network and recurrent neural network, to the boxing movement recognition task and compare the effects with quadratic discriminant analysis and support vector machine. By comparing and analyzing the influence of different network structures on the deep learning algorithm, it is concluded that recurrent neural network has more practical application advantages than graph neural network in network structure parameter tuning.

## 1. Introduction

With the advent of the information age, the human demand for information is increasing day by day. Visual information occupies an important position in the information demand, and the image is the main component of visual information. With the rapid development of electronic technology, there are numerous devices suitable for image information acquisition. Different devices have different degrees of influence on the quality of imaging, while the imaging environment also affects the quality of images [1]. Although good electronic imaging equipment can improve the quality of imaging images, however, because of its high cost and poor universality, that is, different imaging results will appear in different environments, it cannot completely overcome the adverse effects caused by external environmental conditions. In summary, improving image quality does not rely solely on imaging equipment [2]. The digital image processing technology is a series of image processing by the computer so as to achieve the purpose of processing the important part of the original image. In digital image processing, image enhancement techniques occupy an important research position [3]. The image enhancement process can highlight the details of the image and thus improve the clarity of the image. This technique is not only low cost but also highly adaptable, so it is an integral part of image processing technology [4].

In recent years, image reconstruction techniques, as one of the image enhancement techniques, have received attention from many researchers. The goal of image reconstruction algorithms is to enhance low-resolution images to high-resolution images with clear details. Image reconstruction is considered a pathological problem due to the irreversible image degradation process [5]. The reconstructed high-resolution images have different application scenarios depending on the type of image that has been corrupted. High-resolution images contain more detailed information and can effectively support the functional implementation of many computing devices, such as mainframe computers, high-definition TVs, handheld devices, tablets, and cameras [6]. In addition, super-resolution image reconstruction techniques have important applications in static scenes such as target detection (especially small-size object detection), face recognition in surveillance videos, medical image processing, remote sensing imaging, astronomical imaging, and forensic image processing [7].

This paper is divided into five parts: Section 1 provides the research background; Section 2 is the literature review and analysis of the research results of the problem; Section 3 describes the introduction of algorithms related to graph neural networks; Section 4 is a specific experimental analysis of the graph neural network and it shows how the graph neural network performs 3D image reconstruction of sparring action and selects two groups of athletes for comparison; and Section 5 concludes this study.

## 2. Related Works

The following analysis is available for the image reconstruction problem. First, the problem is an inverse problem that does not apply [8, 9]. For reconstructing a high-resolution image from the same low-resolution image, there are multiple solutions rather than a unique solution [10–12]. Therefore, the solution space needs to be reduced based on accurate a priori information. Second, the difficulty of the problem increases when the scaling factor is large. With the interference of complex factors, the image detail information is lost, which makes the reconstruction process more complicated and can lead to the reproduction of error information [13, 14].

Super-resolution image reconstruction methods can be broadly classified into three major categories according to their processing: interpolation-based methods, reconstruction-based methods, and deep learning-based methods [15, 16]. In recent years, deep learning methods have become a booming technology and are growing at an exponential rate, and their performance on super-resolution reconstruction tasks is much higher than that of traditional reconstruction methods [7, 17, 18]. The purpose of deep learning is to automatically learn the relationship between input and output information from data using artificially constructed neural network models under human control [19–21]. Deep learning methods rely on a data-driven approach with training tuning optimization methods to obtain an optimal network model, using which high-resolution images can be reconstructed directly from low-resolution images and the reconstructed images have more detailed information [22]. Although traditional machine learning algorithms can get the desired recognition accuracy in some specific pattern recognition tasks, they suffer from insufficient generalization ability when dealing with some problems with large variations in data features [23]. To address this point, we tried to use deep learning algorithms with stronger generalization ability for classification. Graph neural network (GNN) is a class of efficient classification algorithms that have developed and grown in recent years and has attracted extensive and sufficient attention. In this paper, we investigate the image reconstruction method based on the deep learning method GNN, using the principle of the neural network [24].

## 3. Introduction of Algorithms Related to Graph Neural Networks

### 3.1. Principle of Graph Neural Network Algorithm

This study is centered on the athlete sparring recognition task, which is to determine the current state of the athlete, using pattern recognition methods, by using kinematic or biological information returned from the sensors on the legs. When we perform pattern recognition, the data provided by the sensor is used as input, and the corresponding terrain at this moment is used as output, so this is a supervised learning task and we can use a variety of algorithms including machine learning and deep learning for classification.

In the 1960s, Hubel and Wiesel analyzed the neural structures used for local acuity and directional selection in the cat cortex and learned that their special connectivity structure could efficiently reduce the complexity of information feedback neural network systems, leading to the GNN. The first concrete application of the graph neural network structure was the new discriminator pointed out by K. Fukushima in 1980. Since then, more researchers have improved this model. Among them, the classic model is the “improved cognitive machine” by Alexander and Taylor, which combines the advantages of multiple optimization approaches and avoids the computationally complex backpropagation process.

The leg parameters to be processed in this study have some similarities with speech signals, both of which are classified and recognized as time-series signals. Therefore, borrowing from the way of processing data in speech recognition research, the leg parameters and time series constitute two dimensions of GNN network input data, and the final purpose of classification is achieved through feature extraction of multilayer network structure. The results of the GNN network we mainly used during the experiment are shown in Figure 1.

Among them, layer C represents the convolutional layer, on which multiple convolutional kernels are convolved with the input information of the previous layer to extract common features. The initial weights of the convolution kernels are set randomly, and the weights of the convolution kernels gradually converge to a stable value as the network continuously receives new training data and continuously reduces the cost function through the backpropagation algorithm, which is actually the process of the neural network learning to extract the features of the data itself. In addition to the convolutional kernel weights, the size of the convolutional kernel and the number of convolutional kernels are two parameters that need to be set artificially, which also have a great impact on the final recognition rate. The S layer in the figure represents the pooling layer, which generally alternates with the convolutional layer. The main purpose of this layer is to reduce the dimensionality of the data by pooling the input data from the previous layer, which can reduce the computation and avoid the problem of overfitting the training data that often occurs in deep learning algorithms. The pooling method used in this paper is to divide the data in the previous layer by a certain percentage and then average each piece. Among them, the proportion of division is also one of the adjustable parameters. At the end of the network, this study uses a softmax classifier to map the previously extracted feature information to the gait segmentation.

GNN is a common tool when dealing with sequential data, and the core idea is that whenever a new sample is added, instead of directly reconstructing a new knowledge base, only the information brought by the new sample is adjusted on top of the existing training model. There are many GNN structures, and the most critical point of each structure is how to evaluate the degree of similarity between the new sample and the model in question. This determination criterion affects the way the new samples are subsequently changed for the old database. We used a GNN algorithm designed for intelligent calf legs in our study; this algorithm improved the accuracy of the recognition task across days from 60% to 88.8% in a previous study, but the number of days involved in the experiment for the cross-day test were only two days; we refined and extended on the basis of this study.

### 3.2. Graph Neural Network Automatic Marking

In order to automate the training process, the recognizer first needs to implement automatic pattern identification for the newly completed gait cycle of the leg user. We used in our experiments a dynamic time-based regularization algorithm [38]. This is a tool to determine the similarity of two temporal signals, and it works well when dealing with signals whose length is flexible in the time domain. The results are shown in Figure 2.

The purpose of this method is to *M* match a sequence *X* of a certain length to a template sequence, where the two sequences can be expressed as follows:

(1) $$\begin{array}{c} M=\left(m_{1},m_{2},...,m_{i}\right), \end{array}$$

where *i* ∈ [1, *I*], *j* ∈ [1, *J*], and *x* and *m* are vectors containing 10 channels of IMU information. Define the cost matrix *C* ∈ *R*^*J*×*I*^, where the elements *c*(*j*, *i*)=‖*x*_*j*_ − *m*_*i*_‖^2^. Define the path *P*=(*p*_1_, *p*_2_, ..., *p*_*K*_), where *p*_1_=(1,1), *p*_*k*_=(*J*, *I*), *p*_*K*_=(*j*_*k*_, *i*_*k*_) ∈ [1, *J*] × [1, *I*], and *k* ∈ [1, *K*]; then the total cost of the path P can be expressed as

(2) $$\begin{array}{c} C\left(X,M\right)=\sum_{k=1}^{K}c\left(j_{k},i_{k}\right). \end{array}$$

Furthermore, we calculate the cumulative cost*D*(*X*, *M*) as the cost of the optimal path *P*^*∗*^, with the following expression:

(3) $$\begin{array}{c} D\left(j,i\right)=\min\left\{D\left(j-1,i-1\right),D\left(j-1,i\right),D\left(j,i-1\right)\right\}+c\left(x_{j},m_{i}\right). \end{array}$$

In this study, the sequence *X* ∈ *R*^10×^ denotes F0 the complete gait cycle from one F0 to the next for the same foot, and *J*_*s*_ denotes the number of frames contained in the first *s*_*h*_ gait cycle. A template was constructed M for each of the five movement patterns of each subject, and during the automatic tagging process, the data from the IMU was compared with the template for each complete gait cycle completed by the subject, and the movement pattern corresponding to the smallest cost D(X, M) was automatically tagged, as shown in Figure 3.

### 3.3. Graph Neural Network Template Generation

The template for the class *h* movement pattern for one subject can be calculated by the following equation:

(4) $$\begin{array}{c} t_{m,i}=\frac{1}{K_{i}}\sum_{n=1}^{K}a_{n,i}, \end{array}$$

The first *h* data point is a normalized IMU signal used to generate the number of complete gait cycles of the template and belongs to the first class *h* motion mode. It should be noted that the length of each gait cycle is not a constant value because there will be some differences between each step of the subjects; therefore, in order to ensure that the gait cycle is aligned with the gait cycle in an equal percentage, we use three splines to interpolate the gait cycle *N*_*i*_=*N*_1,*i*_+*N*_2,*i*_. *N*_1,*i*_ and *N*_2,*i*_ denote the number of interpolation points in the swing and support phases, respectively.

### 3.4. Postprocessing of Graph Neural Networks

The data processed by the automatic identification algorithm will be applied to the subsequent classifier retraining, so the accuracy of the identification computed by the dynamic time regularization algorithm is an important factor affecting the recognition effect. In order to reduce the error of automatic identification, we add two methods for data postprocessing after the dynamic time regularization calculation of the data.

First, we compare the DTW results of two adjacent complete gait cycles to see if they are the same, and if they are not; the automatic identification results of the swing phase data that overlap between the two gait cycles are removed from the subsequent model retraining session. The purpose of this is to automatically filter out the data that cannot be classified when gait transitions occur (e.g., from up-kick to flat walk), and it is worth noting that for practical use of the legs, gait transitions generally occur in the swing phase, as shown in Figure 4.

Figure 5 shows a screenshot of the PC interface used to receive the data in the experiment. We will use the pressure sensing information to divide the gait cycle, while the 10 channels of IMU data used in the subsequent analysis include the triaxial acceleration, pitch angle, and roll angle of IMU1 and the triaxial acceleration, pitch angle and roll angle of IMU2.

The experimental scenario is the same as the previous one. In order to examine the effectiveness of GNN and the classifier in the long time period and multiple days of repeated wear experiments, we asked two subjects to do multiple days of experiments, and the number of experimental groups and the number of days between experiments are shown in Table 1. The number of days between adjacent experiments ranged from 1 to 21 days and increased, which was designed to examine the effect of the length of the interval on the recognition effect.

### 3.5. Parameter Setting of Graph Neural Network Classifier

We use a qualifying filter to remove the random pulses from the Euler angles when processing the raw signal acquired by the IMU. If the absolute difference between two adjacent samples is too large and exceeds a threshold, the latter is considered as random noise. The force sensor on the footplate was used to divide a complete gait cycle into two phases: support (stance) and swing (swing), and to define two gait events: foot contact (FC) and foot-off (FO). We segmented the IMU data using a sliding window of 300 ms in length and 10 ms in step length.

In this experiment, we use the QDA, SVM, GNN, and RNN algorithms mentioned in the previous section as classifiers. SVM uses 10 binary classifiers in a one-to-one strategy for the multiclassification task, and the decision model is C-SVC with a polynomial kernel function.

The network structure of the GNN algorithm is as follows: the first hidden layer C1 is a convolutional layer with five convolutional kernels, each with a size of 5 × 2; the second hidden layer S1 is a pooling layer with a pooling ratio of 2 × 1; the third hidden layer C2 is a convolutional layer with eight convolutional kernels, each with a size of 4 × 2; and the fourth hidden layer S2 is a pooling layer with a pooling ratio of 2 × 1.

The RNN algorithm uses an LSTM structure with a 300 ms sliding window and a 10 ms sliding step.

### 3.6. Graph Neural Network Evaluation Method

In this experiment, we still used separate training and testing phases for the swing and stance phases, and the evaluation method used a cross-test between groups. The test group is the data from the first experiment of two subjects, while the training group is the combination of the data from the last five experiments. The recognition error rate is defined as follows:

(5) $$\begin{array}{c} \text{RE}=\frac{N_{\text{mis}}}{N_{\text{total}}}\times 100\%, \end{array}$$

where *N*_total_ denotes the total amount of data contained in the test data set and *N*_mis_ denotes the number of data sets whose classification results do not match the manual markers during the actual test. The recognition accuracy is obtained by subtracting 1 from 1RE.

Since the pattern classification for the terrain recognition task involves multiple modalities, we used the confusion matrix approach in evaluating the recognition effect, whose expression is as follows:

(6) $$\begin{array}{c} R=\left(\begin{array}{ccc} r_{1,1} & ... & r_{1,S}\\ \vdots & \ddots & \vdots \\ r_{S,1} & ... & r_{S,S} \end{array}\right). \end{array}$$

The elements within the matrix are defined as follows:

(7) $$\begin{array}{c} r_{ij}=\frac{s_{ij}}{s_{e}}\times 100\%, \end{array}$$

where *s*_*i*_ denotes the total number of the first *i* motion pattern in the test data and *s*_*i*,*j*_ denotes the number of the first *i* motion pattern identified as the first *j*. Such a representation allows us to examine the recognition relationship between different categories more intuitively. The numerical magnitude of the diagonal elements of the confusion matrix also directly reflects the recognition rate.

Based on the algorithm learning used in the study, the output of the recognizer formed a stream of data and an *N*-point (*N* = 5) majority vote was used to remove random errors. In the postprocessing of the automatic identification, the transition phase was considered successful if the three categories of judgments were correctly labeled as patterned gait events between the first five consecutive outputs of the subsequent motion criticality. In this study, a statistical test for recognition accuracy analysis was performed with a significance level of 0.05.

In our study, we used an automatic marking algorithm based on dynamic time regularization. For this algorithm, we defined the recognition success rate SR as follows:

(8) $$\begin{array}{c} \text{SR}=\frac{N_{C}}{N_{I}}, \end{array}$$

where *N*_*C*_ denotes the number of data sets that are correctly identified automatically using the dynamic time regularization algorithm and *N*_*I*_ denotes the number of all complete step cycles that participate in the automatic identification process.

In the postprocessing process, we also use a threshold *k* value to further improve the accuracy of the automatic identification. The smaller the value of SR, the higher the accuracy SR of dynamic time regularization, but at the same time, the smaller the amount of data involved in template generation. We define the data selection rate DR as follows:

(9) $$\begin{array}{c} \text{DR}=\frac{D_{C}}{D_{I}}, \end{array}$$

where *D*_*C*_ denotes the number of gait cycles for which the distance obtained by the dynamic time regularization algorithm is *C* less than the parameter *k* and *D*_*I*_ denotes the number of all complete gait cycles used in the experiment. In order to obtain a high recognition rate while ensuring an adequate amount of data involved in the automatic marking process, different parameters were tested, and their effectiveness was measured using two metrics, SR and DR.

## 4. Results and Discussion

In previous experiments, the effect of interval days on the training effect could only be assessed by varying the percentage of experimental data within the training set on the same day as the test group, since only two days of experimental data per subject were used as the object of analysis [38]. In this paper, on the other hand, we experimentally collected six days' worth of experiments per subject so that we can examine the effect of the specific value of the number of days of interval on the recognition of motion patterns.

In Figure 6, we can see that the selection of *k* values varies across subjects. We tested the best values for different subjects by using a cross-test between groups in the morning and afternoon on the same day, where the pattern recognition algorithm used was long- and short-term memory. As shown in Table 1, for subject 1, the recognition accuracy SR was 95.6%, and the data selection rate DR was 96.3% when the *k* value was 0.15. Therefore, the value *k* for subject 1 was kept constant at 0.15 in the subsequent experiments. For subject 2, when the value *k* is 0.20, the recognition accuracy SR can reach 92.7%, and the data selection rate DR can reach 94.2%, so the value *k* of subject 2 is chosen as 0.20 in the subsequent experiments.

Since athletes cannot manually label movement patterns during daily exercise, we can use the automatic recognition algorithm described in the previous paper to automatically label newly acquired data. To experimentally validate the effectiveness of this incremental learning strategy, we experimentally simulated the training strategy under leg movements.

The results are shown in Figure 7, where the horizontal coordinate *D*_*i*_ indicates the results of training with the data of the *i*th first experiment and testing with the data of the first experiment. It is worth noting that in this process, we do not use the automatic labeling method for training but use the manual labeling method for training and testing. It can be seen that although the time interval between the experimental set used as the training set and the first experiment kept increasing, there was no significant monotonic trend in the recognition rate, for both subjects. This suggests that the number of days between the data used as the training set and the test data does not have a significant effect on the recognition rate and that the similarity of some environmental factors on the day of the experiment between the training and test sets may have a greater impact.

To test the effectiveness of the automatic identification algorithm in cross-day experiments, we compare the recognition error rates of the two training-testing strategies, and the results are shown in Figure 8, where *T* indicates that the data of one day are used for training and the data of another day are used for testing, while AL indicates that the data of one day are used as a template, the morning (first 24 groups) data of another day are automatically identified, and then the data of the afternoon experiment are tested with the new model. The horizontal coordinate *D*_*i*_ indicates that the *i*th second experiment is used as the training group and the first experiment is used as the test group and corresponds to the T and AL models, respectively. It can be seen from the figure that all recognition error rates decrease after using the automatic marking algorithm. At the same time, the degree of error rate decrease is related to the original high error rate. Taking the result of subject 1 as an example, the highest recognition rate was obtained when using the data of the fifth experiment as the training group, and the recognition rate was improved the most after using the fifth experiment as the template for automatic identification. Therefore, we believe that using the autoidentification algorithm between two groups of data with similar environmental factors can be better for the motion pattern recognition task.

To further validate the effectiveness of the autolabeling algorithm, we compared the training effects of generating groups with different days of data as templates. The results are shown in Figure 9, where T indicates that the ratio of data in the training and test groups is 1:1, no autolabeling algorithm is used, and the training group does not contain data from the same day of the test group. AL1 The morning data in the test group are automatically identified, while the afternoon data are used for testing. It can be seen from the figure that as the amount of data involved in generating the automatic identification template increases, the recognition results are better regardless of the classifier used. For subject 1, compared with other training combinations, when using QDA and GNN for classification, the recognition AL4 error rate decreased the most, even lower than AL5 and AL4. The data added on day 5 are generated as a template, as shown in Figure 7, and the error recognition rate is also the lowest. This shows that adding the experimental group data more matching with the test group to the template generation will greatly improve the recognition effect. The same phenomenon can be seen in Figure 9(b) for subject 2, where the recognition error AL2 rate decreases the most, and the corresponding Figure 7 also shows the lowest error rate for D3 subject 2.

In summary, we can draw the following preliminary conclusions: (1) the length of the interval between the training group and the test group has no significant effect on the accuracy of the recognition task; (2) for the combination of training test results with low recognition rate without automatic identification, the recognition error rate decreases the most after the introduction of automatic identification, and we believe that such a combination has the best matching degree; and (3) when the experimental group with the highest matching degree is added to the template generation library, the recognition effect is most obviously improved when the automatic identification test is done with this template.

## 5. Conclusion

In this paper, the problem of loose hitting in athletes is studied in the following two aspects. We tried to use two deep learning algorithms, graphical neural network and recurrent neural network, in the action recognition task of athletes' sparring and compared them with the effects of quadratic discriminant analysis and support vector machine. After comparing and analyzing the effects of different network structures on deep learning algorithms, it is concluded that recurrent neural networks have more practical use advantages than graph neural networks in terms of parameter tuning of network structures. The performance of four classifiers, namely, quadratic discriminant analysis, support vector machine, graph neural network, and recurrent neural network, in the above-mentioned recognition tasks is then compared and analyzed, and it is concluded that the long- and short-term memory structure (a type of recurrent neural network) can achieve about 95% recognition accuracy in recognition tasks with different data combinations, which is higher than the other three. Support vector machines had the second-highest recognition rate, graphical neural networks the second, and quadratic discriminant analysis the worst.

Based on some of the above conclusions, we also have some perspectives for the future. Ideally, we would like to be able to test the new data by using the usage data of past days as training so as to find out the data of past days with the best match to the new data and use it as a template for automatic identification of the new data. However, in practice, due to the limitation of computing power, we cannot use online real-time training to implement the above strategy. Therefore, on the one hand, we can improve the speed of online training by means of hardware acceleration and parallel computing. On the other hand, we can also try to find a more clever training strategy to make the historical data better support the new data. These are all directions that can be explored in the future.

## Figures and Tables

**Figure 1:** GNN network result graph.

**Figure 2:** Dynamic time-based regularization algorithm.

**Figure 3:** Flowchart of automatic identification.

**Figure 4:** Flowchart of automatic identification postprocessing.

**Figure 5:** Host computer interface diagram.

**Figure 6:** The accuracy of automatic identification under different values of *k*: (a) participant 1 and (b) participant 2.

**Figure 7:** The recognition error rate results of the first experiment as the test group and the training group for the next five experiments.

**Figure 8:** Recognition error rate results of two training and testing strategies: (a) participant 1 and (b) participant 2.

**Figure 9:** The training effect diagram of the group generated by using different days of data as a template: (a) participant 1 and (b) participant 2.

**Table 1:** The number of groups and the number of days between subjects participating in the experiment.

Subjects	*k*	SR	DR
Subject 1	0.15	0.9561	0.9632
Subject 2	0.2	0.9267	0.9417

## Data Availability

The data used to support the findings of this study are available from the corresponding author upon request.
